The article "Design and Application of Major Sports Events Management Information System Based on Integration Algorithm" was published in 2022. Journal: Comput Intell Neurosci.

# Design and Application of Major Sports Events Management Information System Based on Integration Algorithm

**DOI:** 10.1155/2022/6480522

**Published:** 2022-05-16

**Authors:** Yang Wen, Feng Wang

**Affiliations:** ^1^College of Sports Industry and Leisure, Nanjing Sport Institute, Nanjing 210014, China; ^2^School of Physical Education, Taiyuan University of Science and Technology, Taiyuan 030024, China

## Abstract

With the rapid development of social economy and the change of ideology, people are increasingly enthusiastic about participating in sports events. How to make better use of the existing massive network data of sports events to solve the overload of information circulation of sports events has become a potential application problem to promote the development of sports information digitalization. Based on this problem orientation, this paper chooses to study the common characteristics of the current Internet data of sports events and the corresponding and applicable event recommendation technology and constructs feasible event recommendation model as the main direction of solution. The competition information system is the core technology system of the games and the central nervous system of the games. By summing up the previous high-level comprehensive games, the competition information system should serve the competition, command, media, and the public. The smooth construction and stable operation of the perfect design of the competition information system will reflect the organization level of the games and guarantee the success of the games. At the same time, it has certain guiding significance for the design of the competition information system of the large-scale comprehensive games in China in the future.

## 1. Introduction

With the emergence of digital media technology and the popularity of the Internet, In recent years, the sports information work adheres to strengthening top-level design, overall planning, overall benefits of guidelines; each work has made significant progress in information technology and the integration of sports business gradually strengthened, in management and service level, improving the sports industry to promote mass sports and competitive sports development, etc., playing an important supporting role [1–3].

In recent years, with the improvement of China's comprehensive national strength, more and more large-scale sports events are held in China. Large-scale sports events have large scale and long preparation time [4]. It is an extremely complicated systematic project with the characteristics of complex organization and management. Taking the 11th National Games as an example, there will be 33 events, 362 events, 46 delegations, and 12,000 athletes participating in the event. Therefore, it is an inevitable choice to carry out the organization and management of large-scale sports events based on the thought of systems science and the methodology of modern systems engineering and relying on powerful modern science and technology [5]. Major sports events organization and management information system is a kind of integrated use of modern information network and modern digital technology; there will be a large sports organization of internal and external management and service work by optimizing after restructuring to achieve efficient information system tools [6, 7]. By using this system, we can break the restriction of time space and department and provide integrated, efficient, and high-quality information communication services for the smooth holding of large-scale sports events [8].

More and more sports events have become one of the important social and cultural activities. With the increasing social attention and participation, the application of information technology in sports events has become inevitable in the environment of the rapid development of computer information technology. The games competition information system is the core technology system of the games and the central nerve of the games. It can collect, process, and release all kinds of information of the games and serve for the preparation and operation of the games efficiently [9–12]. Effective use of modern information technology means, improving the quality of the work efficiency, to ensure the smooth running of the games, has become an important part of the modern comprehensive games. With the increasing functions and organizational workload of sports events, widely with the public and the news media, information technology also needs to fit modern sporting events of the practical need of the introduction of new design and modern information technology to improve the quality of work [13, 14].

The research of this paper shows that the Internet data of sports events belongs to a part of sports information resources and is fragmented information data [15]. At present, some researches on the application of sports information resources and sports informatization mainly focus on sports information and sports literature, while there is little research on the application of a large number of internet-based fragmented sports event information. In this article, through analysis of the current event information in network, it has the characteristics of the recommendation algorithm to select the appropriate data; the algorithm combined with the data to build a recommended model can be applied to practice matches. It can provide a basis and reference for the application research and related methods of Internet data fragmentation in sports information resources represented by events [16–18]. The second point is to give the possibility of the integration of sports event information and related information technology from the technical perspective, so as to provide a broader idea for the research of sports informatization and enrich the practical significance of the technical means of sports research [1, 19–21].

The contributions of this paper are listed as follows:

1. The recommendation model can be applied to the existing demand of mass competition recommendation, which is a rationalization of demand.
2. The fusion of sports information and technology realized by using recommendation technology and multiple algorithms can also be used to analyze the data information of all the characteristics of relevant events, which has played an essential role in mining and exploring sports data, expanding the application of sports information resources and promoting the fusion of sports and high technology.
3. The application of algorithm in this study to process the feature information of mass competitions can also provide samples and practical reference significance for the integration of sports and other technological formats, which has practical value.

The structure of this article is as follows. The first and second parts give the research status and background. The third part is the design and application of large-scale sports event management information system based on integration algorithm. The fourth part shows the experimental results, and the experimental results are introduced and analyzed with relevant comparison. Finally, the fifth part gives the conclusion of this paper.

## 2. Related Work

There are not many researches on the information technology of large-scale comprehensive sports games [2]. In the process of searching for information, the authors found that many engineering disciplines are involved in the information technology of large-scale comprehensive sports games, but focused on the realization of technology, and the practical application, whether from the point of view of economic benefits or social benefits, could not be implemented [22]. There are several academic studies on the information technology of large-scale comprehensive sports games without focusing on the realization of technology. Li et al. [23] believe that at present China's sports information awareness is not high enough and investment is insufficient. There is no top-level design or relevant technical standards in the system construction as a whole, and the information system construction is at war with each other, unable to connect and share information. Ziakas [24] introduced the competition information system of Beijing Olympic Games in detail and put forward new requirements for the competition information system in the future. They proposed that the information system of comprehensive events should follow four principles: competition as the core, bundled service, balance between stability and advancement, reasonable positioning, and moderate scale. It is the first time that the information system of large-scale comprehensive competition is defined as a service rather than a simple system engineering construction, which is of great guiding significance to the later work [4].

Lei et al. [25] pointed out that the 2008 Olympic Games not only built a huge information system according to the international Olympic Committee (IOC) standard, but also relied on all kinds of open government systems in Beijing, which provided powerful information technology support for the operation of the competition organization of the 2008 Beijing Olympic Games. In recent years, the emergence of the management system has been fundamentally improved from the past human processing affairs, resulting in long cycle, low efficiency, error omission, and other problems [5]. On the basis of the present, the application system with the computer as the carrier emerges in an endless stream. Compared with the previous manual evaluation method, it has made great progress and provides considerable convenience and solves the problems such as large workload, long cycle, low efficiency, and error omission caused by manual operation. In particular, it can solve the problem of clarifying and concreting the process of competition evaluation and making it more convenient to query the results, thus making the management of sports competition more quick, simple, and accurate.

Miles and Shipway [26] concluded from the comparison between the development of sports events and the past that sports events, especially modern sports events, are based on physical movement, constantly challenging the limits of human body, and are the product of civilization and progress of human society. According to Priporas et al. [27], sports events refer to one-time or repeated gathering activities with a certain period of time under the theme of competitive activities, which can have an impact on social economy, tourism development, city reputation, and many other aspects in function. The Internet data of sports events covers both sports events and Internet data at the conceptual level. The concept of sports events studied in this paper has been defined above, while the integration algorithm can be regarded as the information that is displayed and communicated through the Internet platform. Data generally refers to the results that can be obtained through observation experiments or calculation and has various forms such as numerical text and images. This research is based on the Internet technology to build a sports event information exchange storage transmission channel. Taking the 2004 Athens Olympic Games and 2008 Beijing Olympic Games as examples, Esposte et al. [28] concluded that large-scale comprehensive sports events should include timing and scoring, on-site large screen, competition command, TV broadcast, information release, and other systems. However, it should be noted that the weak current facilities of China's stadiums and gymnasiums are basically constructed according to general construction standards, which is difficult to meet the complex needs of future events.

From the above analysis, we know that the above methods have studied the large-scale sports event management information system widely. However, some problems still exist. For example, no scholar has applied the integration algorithm to this field till now, so the research here is still a blank, which has great theoretical research and practical application value for logistics enterprises [29–32], for example, Beijing Olympic Games ticket sales system and event scheduling system.

## 3. Design and Application of Large-Scale Sports Event Management Information System Based on Integration Algorithm

### 3.1. The Structure of Large-Scale Sports Event Management System

The organization management information system of large-scale sports events adopts distributed computing model, and all kinds of organization services are based on communication network and data database service. The system adopts multi-layer architecture, so that the application of the system has greater flexibility and adaptability. On the basis of the lower-level services, specific organization management application modules can be customized for the system. The addition and deletion of some functional application modules do not affect the operation and processing of other parts of the system. For example, the combination of data libraries meets the data requirements of the application layer. The whole system of the method is given in Figure 1.

The system mainly completes the organization and management of human resources in large-scale sports events. The system is responsible for the organization setting and human resources management of the organizing committee, including the recruitment and training of the organizing committee staff and volunteers, personnel assignment, work arrangement, and other management work. The organization and management of human resources in large-scale sports events is to use modern management science to carry out planned recruitment, training, selection, appointment evaluation, and management of employee welfare security, so as to achieve the best allocation of resources. In order to complete the organization and management of logistics support for large-scale sports events, logistics support for large-scale sports events runs through the preparation period of large-scale sports events and the completion period, which is an important guarantee for the success of large-scale sports events. The system is mainly responsible for the organization and management of information communication of large-scale sports events. The system is responsible for the liaison and coordination of sports events and provides relevant services. It collects and manages information, knowledge, and files related to the competition, edits and publishes all kinds of information products, and is responsible for the project approval and approval of publications of the organizing committee. At the same time, the system also includes information consultation of large-scale sports events and organization and management of media reports.

### 3.2. Integration Algorithm

FDA is a supervised discriminant analysis method, and the main idea is to find the optimal projection direction, which maximizes interclass dispersion and minimizes intraclass dispersion. The intraclass dispersion matrix and interclass dispersion matrix are calculated as follows:

(1) $$\begin{array}{c} S^{b}=\sum_{k=1}^{K}n_{k}\left({\bar{x}}_{k}-\bar{x}\right){\left({\bar{x}}_{k}-\bar{x}\right)}^{T}, \end{array}$$

(2) $$\begin{array}{c} S^{w}=\sum_{k=1}^{K}\sum_{x_{i}\in C_{k}}\left(x_{i}-{\bar{x}}_{k}\right){\left(x_{i}-{\bar{x}}_{k}\right)}^{T}. \end{array}$$

In order to introduce LFDA model more conveniently, the equivalent form of FDA algorithm is given on the basis of equations (1) and (2):

(3) $$\begin{array}{c} S_{b}=\frac{1}{2}\sum_{i=1}^{n}\sum_{j=1}^{n}W_{i,j}^{b}\left(x_{i}-x_{j}\right){\left(x_{i}-x_{j}\right)}^{\text{T}}. \end{array}$$

And

(4) $$\begin{array}{c} S_{w}=\frac{1}{2}\sum_{i=1}^{n}\sum_{j=1}^{n}W_{i,j}^{w}\left(x_{i}-x_{j}\right){\left(x_{i}-x_{j}\right)}^{\text{T}}. \end{array}$$

And the weight calculation is as follows:

(5) $$\begin{array}{c} W_{i,j}^{w}=\left\{\begin{array}{cc} \frac{1}{n_{k}} & \text{if }x_{i},x_{j}\in C_{k},\\ 0 & \text{others.} \end{array}\right)n \end{array}$$

And

(6) $$\begin{array}{c} W_{i,j}^{b}=\left\{\begin{array}{cc} \left(\frac{1}{n}-\frac{1}{n_{k}}\right) & \text{if }x_{i},x_{j}\in C_{k},\\ \frac{1}{n} & \text{others.} \end{array}\right.\\ a_{u,v}^{\left(l\right)}=f\left(z_{u,v}^{\left(l\right)}\right). \end{array}$$

The projection direction of the LFDA model can be obtained by solving the following equation:

(7) $$\begin{array}{c} J_{\text{LFDA}}=\underset{\hat{w}}{\text{argmax}}\frac{{\hat{w}}^{\text{T}}{\hat{S}}^{b}\hat{w}}{{\hat{w}}^{\text{T}}{\hat{S}}^{w}\hat{w}}. \end{array}$$

For the new test data set *X*, it can be divided into specific categories by the following discriminant function:

(8) $$\begin{array}{c} g_{k}\left(x\right)=-\frac{1}{2}{\left(x-{\bar{x}}_{k}\right)}^{\text{T}}T_{r}\Gamma^{-1}T_{r}^{\text{T}}\left(x-{\bar{x}}_{k}\right)+\mathrm{In}K-\frac{1}{2}\mathrm{In}\left[\det\left(\Gamma \right)\right],\\ \Gamma =\frac{\left(T_{r}^{\text{T}}\left[\sum_{x\in C_{k}}\left(x-{\bar{x}}_{k}\right){\left(x-{\bar{x}}_{k}\right)}^{\text{T}}\right]T_{r}\right)}{n_{k}-1}. \end{array}$$

Since different variable quantum blocks may have different effects on fault classification, in order to better depict the differential effects of different subblocks on diagnosis results, the following integrated discriminant function is established by using weighting strategy:

(9) $$\begin{array}{c} Ig_{k}\left(x\right)=\sum_{l=1}^{M}w_{l}g_{k}^{\left(l\right)}\left(x\right). \end{array}$$

The weight matrix is defined as follows:

(10) $$\begin{array}{c} w_{l}=\frac{{\hat{w}}_{l}}{\sum_{l=1}^{M}{\hat{w}}_{l}}\;{\hat{w}}_{l}={\left({\text{Acc}}_{l}\right)}^{2}. \end{array}$$

From the above analysis, if the classification accuracy of training data in a subblock is higher, the weight coefficient of the subblock will be higher, and its function in the integrated model will be more important, and vice versa. The ILFDA model can describe the local characteristics of data from two dimensions of sample and variable, highlight the role of sample local information and variable local information in fault classification more comprehensively, and help improve the accuracy of fault classification. The schematic diagram of a typical convolutional neural network is shown in Figure 2.

This system mainly completes the large-scale sports event marketing organization and management and is responsible for large-scale sports events sponsorship, advertising, ticket sales, media, business license sales, raise fund raising, public relations, courtesy, consumers, target marketing, product segmentation, marketing price, sales promotion market research, marketing plan, sales of intangible assets, media, and PR. Large-scale sports competition management is the core work of large-scale sports event organization management. All the organization and management activities are for the management of large-scale sports events. Competition management of large-scale sports events is jointly participated by competition managers, athletes, referees, spectators, volunteers, news media, and other participants of sports events. The essence of competition organization and management of large-scale sports events is to manage the competition activities of large-scale sports events, effectively improve the quality of sports events products, and achieve the goals and objectives of sports events.

## 4. Experimental Results and Analysis

### 4.1. Introduction to Experimental Environment and Data Set

This line of business was on Windows 11 OS runs a HMP RTX 2070S 8 GB video memory, AMD Ryzen 2400G CPU, 8 GB DDR4 software environment: deep learning framework PyTorch 1.7. Python 3.8 CUDA 10.0.

### 4.2. Experimental Results Analysis

Firstly, the comparison of the results of the sport data analysis chart under different time is given in Figure 3. After the modeling of the event recommendation model through the above process, it is necessary to compare the sports data of each algorithm model under the same conditions. According to the evaluation method of this experiment, it can be seen that the recommendation accuracy of calculating the event recommendation model is related to the length of the list of events to be recommended and the categories of events browsed by users. Therefore, the length of the list of events to be recommended should be unified during the experimental evaluation.

In this experiment, the value range of the list length of the event to be recommended was used to observe the recommendation accuracy of the event recommendation models with different algorithms under the change of the list length. In the experimental results, the accuracy of the event recommendation model of different algorithms is the corresponding variation line graph, indicating the recommendation performance of the event recommendation model of different key algorithms under different input sample data sets.

It can be seen from Figure 4 that the data loading efficiency of network interface in system is different. The comprehensive recommendation model based on HTTP text weight model and OMI series has excellent performance, and the overall recommendation accuracy is about 80%. When the length of the recommendation list is 10 or larger, the recommendation performance is stable and the recommendation accuracy is above 77%. Compared with the content recommendation model based on a single algorithm, the comprehensive content recommendation model can achieve better recommendation performance, and it also verifies that the comprehensive event integration model proposed in this paper has advantages in performance. However, the event recommendation models based on three different single algorithms are different in recommendation performance.

Among them, the algorithm based on o-DF sequence model has a good recommendation performance on the Internet data set of sports events. The number of recommendation lists tends to be stable within [7, 26], and the recommendation accuracy is stable at more than 72%. When the length value of the recommendation list is less than 7, the recommendation instability is easy to occur. The reason may be that there is a difference between the user's implicit selection feature mined by o-DF sequence model and the user's displayed selection feature, which belongs to the instability of the algorithm model. It can be seen that, in the actual event recommendation target, the existence of user participation sequence data can better mine the association between users and the event. In the case of a large number of recommendations to be made, a single model is difficult to achieve a good recommendation effect.

Figure 5 shows management efficiency of sports events before and after optimization. The selection of system modules should take into account the needs of special projects of comprehensive sports events and the host city, as well as the operation and management requirements of all departments of the organizing committee. However, it is suggested that the management system should be reused as far as possible, and the development and construction should be started after special needs, so as to better deal with post-game information assets. Operation guarantee is a problem to be considered as a system designer. The schedule should be designed and arranged in advance, reasonably planned in the form of inverted time, and enough time should be reserved for the required actions such as testing and joint adjustment, so that the combination of advanced technology and subsequent matching operation can ensure the complete functional presentation of the large-scale comprehensive games information system. So we need to optimize and upgrade the system.

As shown in Figure 6, we can also see the changes in the efficiency and satisfaction of event management before and after the optimization of the system. It can be seen that, after optimization, satisfaction and management efficiency are improved with the increase of the number of matches. Therefore, it is necessary to optimize the analysis system of large-scale competitions.

According to statistics, there are 4944 event information in the collected data set, among which 2912 event records have been recorded in the recent three years from 2017 to 2019, which also reflects the booming development of marathon and road running in China in recent years. Statistical description of event data volume is no longer divided into individual years. Among them, there are 617 events with more than 100 participants and 497 events with more than 100 followers. The maximum values of the two events both appear in the data set of Shanghai International Marathon; the top three regions with the most event records are Zhejiang, Jiangsu, and Shanghai, with 611, 516, and 427 events, respectively. A total of 979 events with recorded information have been held in these three regions from 2017 to 2020. It can be seen that the Yangtze River Delta region is the most active region for marathon and road running events in recent years. There are 457 overseas events covering 80 countries and regions, among which the United States region has the most recorded data of 110 events in total.

In the data table of competition information, there are 56,057 valid users with 264,079 entries. The average user has participated in about 4.71 events, among which the runner user has the largest number of entries and has participated and recorded 130 marathon events in total. The users who participated in the event in the data collection were classified and counted as having participated in the event for 3 times and less than 3 times and less than 10 times and more than 10 times and less than 20 times and more than 20 times. The results are shown in Figure 7. More than half of the users who participated in the race for 3 times or less and the users who participated in the race for more than 10 times accounted for less than 10% of the total, indicating that a large number of runners in this data set did not participate in the race for many times. Professional marathon runner users belong to a very small portion of this user cluster.

As shown in Figure 8, we can see the structure of the actual record of the competition in the system, and the system can record all kinds of information in the competition intuitively and clearly. Modular design of the system in each subsystem coupling degree is low, can be decomposed, and can be combined advantages, The modules of the system are easy to understand, and the system can be split and combined according to the actual needs of large-scale comprehensive events held in China in the future to form a suitable event information system. In addition, the scheme design adopts a standardized design mode internally, but there is no standard basis externally. From the policy level to promote the standardization of sports information technology, this is one of the directions that needs to continue efforts in the future.

## 5. Conclusions

Based on the data analysis and expert interviews of the competition information system of comprehensive sports events for many years, combined with the actual operation process of the games, the study determined that the selection of system modules, operation guarantee, risk supervision, and control constitute three necessary steps for the design of the competition information system of large-scale comprehensive sports events. It can provide relevant planning suggestions for the subsequent design of the competition information system of large-scale comprehensive sports events. The selection of system modules should take into account the needs of special projects of comprehensive sports events and the operation and management requirements of various departments of the organizing committee of the host city. However, it is suggested that the management system should be reused as far as possible, and the development and construction should be started after special needs, so as to better deal with post-game information assets.

Risk monitoring is a problem that must be considered for many large-scale activities, especially for influential projects such as the people's games; there are many professional researches on risk analysis and response, which need to be advanced over time. Using advanced tools and technologies to reduce the risks of the games is also a worthy direction of future research.

## Figures and Tables

**Figure 1:** Structure of large-scale sports event management system.

**Figure 2:** The schematic diagram of convolutional neural network.

**Figure 3:** Sport data analysis chart.

**Figure 4:** The data loading efficiency of network interface. (a) Data load (bytes) and efficiency ratio of the web interface. (b) Data load (bytes) and efficiency ratio of the REST interface (HTTP GET). (c) Data load (bytes) and efficiency ratio of the REST interface with O-DF payload (HTTP POST).

**Figure 5:** Management efficiency of sports events before and after optimization.

**Figure 6:** Different methods for recoloring gray image.

**Figure 7:** The classification of user participation times.

**Figure 8:** Example of timing plate. (a) The rest of the timing plate. (b) Timing plate match.

## Data Availability

The data used to support the findings of this study are available from the corresponding author upon request.
